The article "CT Image Examination Based on Virtual Reality Analysis in Clinical Diagnosis of Gastrointestinal Stromal Tumors" was retracted in 2023. Reasons: signs of a paper mill; suspected computer-generated content; unreliable results or conclusions; lack of ethics approval or compliance.

# CT Image Examination Based on Virtual Reality Analysis in Clinical Diagnosis of Gastrointestinal Stromal Tumors

**DOI:** 10.1155/2021/9996565

**Published:** 2021-06-16

**Authors:** Zhiying Wang, Qiaoyan Qu, Ke Cai, Ting Xu

**Affiliations:** ^1^Department of Gastroenterology, West District of Qingdao Municipal Hospital, Qingdao 266000, Shandong, China; ^2^Internal Medicine, Songshan Hospital of Medical College of Qingdao University, Qingdao 266000, Shandong, China

## Abstract

With the advancement and development of medical equipment, CT images have become a common lung examination tool. This article mainly studies the application of CT imaging examination based on virtual reality analysis in the clinical diagnosis of gastrointestinal stromal tumors. Before extracting suspected lymph nodes from a CT image of the stomach, the CT image sequence is preprocessed first, which can reduce the cumbersomeness of subsequent extraction of suspected lymph nodes and speed up the subsequent processing. According to medical knowledge, CT images of the stomach show that lymph nodes mainly exist in the adipose tissue around the gastric wall, but there are no lymph nodes in the subcutaneous fat outside the chest. The most basic gray value in the image and the neighborhood average difference feature related to gray level are used as the primary features of visual attention detection. When extracting the neighborhood average difference feature, we use a 3^*∗*^3 sliding window method to traverse each point of the pixel matrix in the image, thereby calculating the feature value of each pixel in the image. After the feature extraction is completed, it is necessary to calibrate the data and make a training data set. The SP immunohistochemical staining method was used. The specimens were fixed with 10% formaldehyde, routinely embedded in paraffin, sectioned, and stained with HE. The tumor tissue was determined by immunohistochemistry, and the reagents were products of Maixin Company. All patients were followed up by regular outpatient review, letters, and visits or phone calls. The data showed that immunohistochemical tumor cells showed positive staining for CD117 (14/15, 93.3%) and CD34 (10/15, 66.7%). The results show that the application of virtual reality technology to CT imaging examination can significantly improve the diagnostic accuracy of gastrointestinal stromal tumors.

## 1. Introduction

At present, the clinical application of multilayer CT is in a large-scale promotion stage in China, and many basic hospitals have introduced multilayer CT. The CT Department of grassroots hospitals has the characteristics of less diagnostic doctors, less computer equipment, and general configuration. The number of patients in these CT departments is large every day, which is more than the resources that can be used in clinical diagnosis. In essence, virtual reality technology is an advanced computer user interface. It provides users with various intuitive and natural real-time perception and interaction methods such as viewing, listening, and touching at the same time, so as to maximize the convenience of users' operations, reduce the burden on users, and improve the efficiency of the entire system.

For the diagnosis of gastrointestinal stromal tumors, the computer-aided detection of lymph nodes near the stomach is particularly important because the morphological changes and metastasis of gastric lymph nodes are the wind vane for doctors to diagnose gastrointestinal stromal tumors, and the analysis of lymph nodes near the cancer focus can help doctors more accurately determine the lymph node staging of patients, predicting the metastasis mechanism and determining the future treatment plan can strive for greater survival rate for patients. Because the determination of the lesion depends on the subjective observation and judgment of the doctor to a great extent, it not only increases the workload of the doctor and puts forward high requirements for the professional quality of the doctor, but also leads to all kinds of misdiagnosis.

Virtual reality technology has been widely used in various fields. Mahawongkajit et al. believe that thorough surgical resection is essential for the permanent cure of patients with gastrointestinal stromal tumors (GIST). Laparoscopic wedge resection is a widely accepted surgical treatment method, but when using this technique, it is a challenge to identify tumor margins from the perspective of serosal laparoscopy. Nonexposure endoscopic inversion (NEWS) for patients with gastric GISTs is a novel minimally invasive surgical technique that can assist in the complete resection of tumor margins through endoscopic and laparoscopic methods, remove the entire stomach wall and the entire tumor, and reduce the risk of peritoneal contamination or tumor spread to the peritoneum. A computed tomography scan accidentally found a gastric mass protruding into the lumen. Although their research has certain feasibility, it lacks specific experimental content [1, 2]. Rausch et al. believe that most gastrointestinal stromal tumors (GISTs) are caused by activated mutations of kit receptor tyrosine kinases. Imatinib mesylate, a small molecule inhibitor, was initially developed to target abl1 kinase, which is constitutively activated by chromosome translocation in BCR-ABL1 positive chronic myeloid leukemia. Imatinib has been successfully used in the treatment of GIST due to its cross reactivity with kit kinase. Although inhibition of kit obviously plays a major role in the therapeutic response of gist to imatinib, the concomitant inhibition of ABL in this case has never been explored. Although his research is more accurate, it lacks necessary experimental data [3]. Yin and Zhang believe that gastrointestinal stromal tumors (GIST) are the most common gastrointestinal stromal tumors. Any medical exploration and practice is originally designed to have the essence of humanism. In addition, doctors should comprehensively consider the patient's physical, psychological, and social attributes, pay attention to the patient's physical, psychological, and social needs, and find and try to solve problems, so as to promote the development of medical science in the right direction. Although their research is relatively comprehensive in theory, it lacks a specific operation plan [4]. Cao and Wang believe that gastrointestinal stromal tumors (GIST) are the most common stromal tumors in the gastrointestinal tract. They analyzed the pitfalls and misunderstandings in all aspects of GIST diagnosis and treatment and provided clues for promoting more reasonable clinical decision-making. Although their research has a certain positive effect, there are still many loopholes [5, 6].

The diagnosis of gastrointestinal stromal tumor largely depends on the lymph node metastasis of gastrointestinal stromal tumor. In order to realize the early diagnosis and treatment of gastrointestinal stromal tumor and reduce the mortality of gastrointestinal stromal tumor, it is necessary to design a method that can quickly and effectively detect lymph nodes from gastrointestinal stromal tumor to help professional doctors make further diagnosis. Aiming at the problem of lymph node detection in gastrointestinal stromal tumors, combined with the relevant knowledge of image processing and pattern recognition, this paper designs a lymph node detection framework; using image processing methods to detect regions of interest from CT images, extract suspected lymph nodes, and then combine the target based on the tracking related knowledge, the lymph nodes can be extracted based on the status information of the suspected lymph nodes on the sequence images.

## 2. Virtual Reality Analysis and CT Imaging Examination

### 2.1. Virtual Reality Technology

Virtual reality technology digitizes and directly reappears the product scheme from 2D drawings and 3D models, mimics the shape, color, material, size, and other attributes of the product, and provides a digital product that can be viewed and used in virtual world for evaluation and verification of evaluators. Virtual reality technology can not only simulate the appearance of products with high precision, but also build the environment for product use and simulate the process of product use. Through strong technical support, the appraisers can observe and use the products in the realistic and natural and reasonable use environment and make the evaluation results more reasonable [7].

The entity and the virtual body are inseparable, and the dialectical relationship between the two constitutes the product and determines the grade of the product. On the one hand, the two are related to each other. The virtual body belongs to the ideology. It cannot exist in isolation. It must be based on the entity. That is to say, the product materials, design tools, related processing equipment, etc. must be considered in the design process and whether to support the completion of product manufacturing. Moreover, the perceptual elements of the product need to be externalized by the product entity [8, 9]. In addition, human beings live in a real environment, surrounded by objective entities. Objective entities are the necessities of human life, and the real sense of human existence needs to be reflected by product entities. On the other hand, the two restrict each other. The perfection of the physical elements directly restricts the degree of manifestation of the virtual elements. Without physical support, regardless of unique creativity, that is, no matter how beautiful ideas can be realized, excellent products cannot be realized [10].

According to the rough set theory, assuming that *R*={*C*_1_, *C*_2_,…, *C*_*n*_} is the evaluation result set of *n* persons, then

(1) $$\begin{array}{c} \underline{{\text{Apr}}_{C_{i}}}=\cup \left\{C_{k}\leq C_{i}\right\},\;k=1,2,\ldots ,n, \end{array}$$

(2) $$\begin{array}{c} \bar{{\text{Apr}}_{C_{i}}}=\cup \left\{C_{k}\geq C_{i}\right\},\;k=1,2,\ldots ,n. \end{array}$$

The fuzzy number of *C*_*i*_ is

(3) $$\begin{array}{c} RN_{C_{i}}=\left[C_{i}^{L},C_{i}^{U}\right], \end{array}$$

(4) $$\begin{array}{c} C_{i}^{L}=\frac{\sum \underline{{\text{Apr}}_{C_{i}}}}{M_{L}}, \end{array}$$

(5) $$\begin{array}{c} C_{i}^{U}=\frac{\sum \bar{{\text{Apr}}_{C_{i}}}}{M_{U}}. \end{array}$$

Among them, *M*_*L*_ represents the number of the lower limit of *C*_*i*_, and *M*_*U*_ represents the number of the upper limit of *C*_*i*_ [11].

The use of virtual reality technology can simulate a variety of city models, so as to deeply analyze the spatial, temporal, and attribute information of digital city, and promote the application of digital city to a higher level. The use of virtual reality technology can make people see the face of the city after the design and adjust the line of sight according to the spatial location and size. Virtual reality expands the virtual environment and creates a virtual space. It presents the city in an intuitive, three-dimensional graphic environment in front of people, replacing the traditional abstract map and descriptive documents used to explain, analyze, and discuss design ideas and urban development [12, 13]. In VR environment, the operator can freely choose the motion mode and trajectory and determine the observation height, motion speed, and other related parameters. In this way, architects can consider more factors in the design and take into account different levels, so that the designed works are closer to life, more natural and more scientific [14].

### 2.2. CT Imaging Examination

Traditional CT, MRI, US, and other imaging equipment can only show the size, shape, density, and other pathological features of the tumor and the relationship with surrounding tissues, can only provide anatomical and morphological information, internal microenvironment cannot be distinguished, and accurate diagnosis cannot be made. CT imaging is currently the most common high-quality medical image. It is a digital expression of human cross-sectional information [15]. Each CT image is composed of a certain number of pixels, and what each pixel reflects is the CT value information corresponding to the human tissue at the coordinate position. After the rays passing through the tissue reach the detector, if the number of attenuated rays is sufficient, they are sent to the computer to reconstruct the image; if not enough, the X-ray irradiation time needs to be lengthened [16].

Let the window width be *W* and the window level be *L*; the CT value is *v*, the gray value is *g*, and 0 ≤ *g* ≤ 255. The specific form of the piecewise function is

(6) $$\begin{array}{c} g=\left\{\begin{array}{cc} g_{\min}, & v<\left(L-\frac{W}{2}\right),\\ g_{\min}+\frac{v-\left(L-W/2\right)}{W}\times \left(g_{\max}-g_{\min}\right), & \left(L-\frac{W}{2}\right)\leq v\leq \left(L+\frac{W}{2}\right),\\ g_{\max}, & v>\left(L+\frac{W}{2}\right). \end{array}\right. \end{array}$$

The indicators for evaluating the quality of the segmentation results are overlap (Overlap) and mismatch (Mismatch). *R*_gold_ and *R*_new_ refer to the standard pixel set and the pixel set of the segmentation algorithm, respectively.

(7) $$\begin{array}{c} \text{overlap }={\frac{R_{\text{gold}}\cap R_{\text{new}}}{R_{\text{gold}}\cup R_{\text{new}}}}^{*}100\%, \end{array}$$

(8) $$\begin{array}{c} \text{mismatch }=\;{\frac{R_{\text{gold}}\cup R_{\text{new}}-R_{\text{gold}}\cap R_{\text{new}}}{R_{\text{gold}}}}^{*}100\%. \end{array}$$

The fitness function can be described as the sum of the square error criterion function; the expression is as follows:

(9) $$\begin{array}{c} J\left(M\right)=\sum_{j=1}^{N}\min\left(D_{1j},D_{2j},...,D_{kj}\right),\;i=1,...,k,\;j=1,...,N. \end{array}$$

In the formula, *D*_*ij*_ is the distance from the *i*th cluster center to the *j*th sample in the feature space. Specifically, the CT image is that the transmitted rays pass through the imaged human tissue in a specific way. The rays passing through the human body are received by the detector and converted into digital signals according to their attenuation degree, which is processed by the computer to form a cross-sectional image of the human body. After the rays passing through the tissue reach the detector, if the number of attenuated rays is sufficient, they are sent to the computer to reconstruct the image; if not enough, the X-ray irradiation time needs to be lengthened [17].

The characteristic value is

(10) $$\begin{array}{c} f_{1}=\left|g\left(p\right)-g\left(q\right)\right|, \end{array}$$

(11) $$\begin{array}{c} f_{2}=\frac{1}{3}\left|g\left(p\right)+g\left(t\right)+g\left(v\right)-g\left(q\right)-g\left(u\right)-g\left(w\right)\right|, \end{array}$$

(12) $$\begin{array}{c} f_{3}=\frac{1}{2}\left|g\left(p\right)+\frac{1}{2}g\left(t\right)+\frac{1}{2}g\left(v\right)-g\left(q\right)-\frac{1}{2}g\left(u\right)-\frac{1}{2}g\left(w\right)\right|, \end{array}$$

(13) $$\begin{array}{c} f_{4}=\frac{1}{4}\left(\left|g\left(p\right)-g\left(u\right)\right|+\left|g\left(t\right)-g\left(q\right)\right|+\left|g\left(p\right)-g\left(w\right)\right|+\left|g\left(v\right)-g\left(q\right)\right|\right). \end{array}$$

The feature conversion function is

(14) $$\begin{array}{c} c_{1}\left(f\right)=\left\{\begin{array}{cc} 1, & f\leq l_{1}+\frac{a^{2}}{2},\\ \frac{a^{2}}{2\left(f-l_{1}\right)}, & l_{1}+\frac{a^{2}}{2}<f\leq l_{2},\\ 0, & f>l_{2}. \end{array}\right. \end{array}$$

Among them, *a*, *l*_1_, and *l*_2_ are free parameters.

By carefully observing each frame of CT images, combined with a series of multiframe image observations, a dynamic visual angle can be used to intuitively sense the internal information of organs and tissues. The ability to visualize the area to be inspected on the CT image is a magic weapon for the doctor to successfully diagnose. In the CT image, as long as the pathological area is large enough and other areas that are close to the same have a large grayscale difference, then this time it can be developed correctly [18, 19].

### 2.3. Gastrointestinal Stromal Tumors

The imaging findings of gastrointestinal stromal tumor are shown in Figure 1. The four corners of the image are divided by a circle. If the corners are selected as the seed points for region growth, it is necessary to use the four corners to process the region growth algorithm separately. Since the size of the stomach CT image is 512 × 512, and the stomach parenchyma is always in the middle part of the image, use these pieces of prior knowledge to directly draw a suitable ring on the image to keep the edges and corners of the image connected [20].Tumor metastasis is a multistep and complex process. Tumor cells need to complete a series of biological processes when they migrate from the primary tumor to specific tissues and organs to form metastasis, among which angiogenesis, matrix degradation, and tumor cell adhesion and colonization are the most important. In human tissues, a variety of cytokines and proteins are involved in the process of tumor metastasis [21].

The ultrasound images of liver GISTs showed intrahepatic hypoechoic images, most of the tumors had clear boundaries, and some blood flow signals were visible. The significance of ultrasound examination for liver GISTs lies in the discovery of lesions and preliminary judgment of the nature of the tumor. Because it can repeatedly observe the shape, size, and quantity of the tumor, it has a certain value in judging the nature of the tumor. Surgical methods are divided into surgical radical resection and palliative resection [22].

Biological behavior judgment refers to GIST. The pEGIST risk grades in this group are all high risk. Among them, 2 cases of tumor ruptured, and the number of mitoses was greater than or equal to 10/50 HPFs, and most tumors were more than 10 cm in diameter; tumor rupture indicated a high possibility of recurrence and metastasis. Therefore, EGIST often presents a high degree of risk. Tumors in this group located outside the gastrointestinal tract are often misdiagnosed by clinicians. For example, the pelvic region is easily misdiagnosed as leiomyoma or leiomyosarcoma; the latter is easily misdiagnosed as dedifferentiated liposarcoma, fibrosarcoma, and other soft tissue sarcomas when it occurs in the peritoneum. However, due to lack of clinical understanding, tumors often fail to receive correct treatment and often lead to recurrence [23, 24].

## 3. Clinical Diagnosis Experiment of Gastrointestinal Stromal Tumor

### 3.1. Subjects

Select 300 patients diagnosed with gastrointestinal stromal tumors and establish a database. The clinical data collected include age, gender, chief complaint or symptoms, imaging examinations, surgical records, tumor rupture, and postoperative imatinib treatment. The collected pathological data include tumor size, tumor location, histological type, mitotic number, risk grade, tumor necrosis, immunophenotype (CD117, DOG-1, CD34, and Ki-67), and tumor and surrounding tissues relationship [25, 26].

### 3.2. Experimental Equipment and Reagents

The main instruments used in the experiment are dehydrator, dyeing machine, slicer, automatic immunohistochemical dyeing machine, low-temperature refrigerator, high-temperature pressure steam sterilizer, electric-heating constant-temperature blast drying oven, etc.; the main reagents are CD117, D0G1, CD34, S-100, SMA, etc. [27].

### 3.3. CT Imaging Examination

Before extracting suspected lymph nodes from a CT image of the stomach, the CT image sequence is preprocessed first, which can reduce the cumbersomeness of subsequent extraction of suspected lymph nodes and speed up the subsequent processing. According to common medical knowledge, observing the CT images of the stomach, the lymph nodes mainly exist in the fat tissues around the stomach wall, while the subcutaneous fat outside the thoracic cavity does not contain lymph nodes. The tumor size is defined as the maximum diameter of the tumor, and the mitotic figures are defined as the number of mitotic figures per 50 times high-power field of view. The diagnosis of patients with metastasis is based on imaging examinations (such as CT, MRI, B-ultrasound, etc.) or pathological puncture. They are divided into only liver metastasis group and only abdominal and pelvic implant metastasis group [28, 29].

### 3.4. Feature Extraction

The most basic gray value in the image and the neighborhood average difference feature related to gray are used as the primary features of visual attention detection. When extracting the neighborhood average difference feature, we use a 3 ^*∗*^3 sliding window method to traverse each point of the pixel matrix in the image to calculate the feature value of each pixel in the image [30]. This article saves the areas to be inspected in the form of a file, and each area to be inspected is a folder, which contains images of three faces and a text. The location information is recorded in the data [31].

### 3.5. Judgment of Positive Immunohistochemistry Standard

The SP immunohistochemical staining method was used. The specimens were fixed with 10% formaldehyde, routinely embedded in paraffin, sectioned, and stained with HE. The tumor tissue was determined by immunohistochemistry, and the reagents were products of Maixin Company. Each case was stained with CDI17 and CD34. Among them, CD117 is envision kit, and CD34 is SP kit. Regardless of the intensity range of SP staining, the tumor cells with cytoplasmic brown particles can be judged as positive [32].

### 3.6. Follow-Up

The survival status of patients was followed up by telephone and letters. All patients were followed up by regular outpatient review, letters, and visits or telephone calls. The evaluation of treatment-related adverse reactions is carried out monthly, and the evaluation method is to recheck blood routines, liver and kidney function, and other blood tests and conduct toxic and side effects evaluation [33].

### 3.7. Statistical Processing

All parameters were processed by SPSS15.0 statistical software. Chi-square test was used for univariate analysis of survival rate, and COX regression model was used for multivariate survival analysis. Survival rate was calculated by direct method. Tumor diameter was expressed as mean and standard deviation. The results are presented in the form of percentage or median (range), and Kaplan–Meier method is used to generate a survival curve [34].

## 4. Results and Discussion

### 4.1. Clinicopathological Analysis

The ultrasound appearance of gastrointestinal stromal tumors is shown in Figure 2. For CT sequence images, the gastric nodules are detected and extracted first, and then the sagittal and coronal reconstructions are performed on the area extracted by the detection, and the features of the area to be recognized are calculated and extracted from the three view planes, and the features are normalized and the chemical processing is input to the trained model, and the classification model is the output of the classification and recognition results. In short, this algorithm introduces wavelet denoising method in the processing process, which can effectively remove Gaussian white noise and random noise, and the resulting image is clearer. At the same time, the entire transformation process revolves around the edge features of the image, which effectively protects and enhances the edge features of the image, and highlights the most valuable information in the CT image. Finally, the exponential and histogram equalization transformation is performed on the CT image, and the gray level of the region of interest is adjusted, so the overall characteristics of the image are improved and the outline is clearer.

The test time comparison is shown in Table 1. The virtual reality CT detection algorithm proposed in this paper has an average detection time of 5.1 s in CT images; it saves 2.35 s compared with the traditional random forest detection algorithm and 15.72 s compared with the AdaBoost detection algorithm. Improved GA can get better results than traditional GA when using a smaller number of features. It is further verified that if the features in the feature set are independent of each other, the more the number of feature sets, the better the recognition effect. In the clinic, we try to integrate the overall situation of the patient as much as possible. For patients who can undergo surgery, we can achieve RO resection as much as possible. For patients with extensive liver metastasis or unable to undergo RO resection, targeted therapy should be performed before surgery. When targeted therapy can completely shrink the tumor, resection is performed at this time.

The main characteristics of gastrointestinal stromal tumors are shown in Figure 3. The diameter of the patient's tumor was between 5 and 27 cm, with a median diameter of 12.0 cm. The microscopic findings: spindle cells (12/15, 80%), spindle cells-epithelial-like cells mixed (4/15, 20.0%), and mitotic figures (13/15, 86.7%) > 5/50 HPF. Immunohistochemistry tumor cells showed positive staining for CD117 (14/15, 93.3%) and CD34 (10/15, 66.7%). Tumor cells of the spindle cell type are composed of short spindle to elongated spindle cells arranged in a spiral, fence, or bundle. The cytoplasm of the tumor cells is less, the cytoplasm is red or lightly stained, and the nucleus is spindle-shaped. When the nucleus is dark, small nucleoli are occasionally seen, and in some tumor cells, vacuoles can be seen at the end of the nucleus, nuclei have different degrees of atypia, and the number of mitotic figures is different in different cases.

The multivariate COX regression analysis of the postoperative survival rate of patients is shown in Table 2. Among them, gastric stromal tumors have the best prognosis, with a 3-year survival rate of 59.3%, and the worst in the small intestine (24.2%). The high postoperative survival rate (80%) of colorectal stromal tumors may be related to the small number of cases and large errors. Tumors with small diameter and no recurrence and metastasis after surgery have a good prognosis.

The multifactor analysis of risk factors in the abdominal and pelvic implant transfer group is shown in Table 3. The results of multivariate analysis showed that tumor diameter > 10 cm and ascites were the risk factors of abdominal and pelvic metastasis. The c-kit gene mutation rate of gastrointestinal stromal tumors was 88.2% in spindle cell type, 60.0% in epithelial cell type, and 61.9% in mixed cell type. There were significant differences in the c-kit gene mutation rate among different tissue types of gastrointestinal stromal tumors (*p* = 0.002). The mutation rate of c-kit gene in spindle cell type was higher than that in epithelial cell type (*p* = 0.033) and mixed cell type (*p* = 0.006). The mutation rate of c-kit gene in very-low-risk group was significantly lower than that in low-risk group (*p*= 0.022), medium-risk group (*p* = 0.006), and high-risk group (*p* = 0.009). There was no significant difference in the mutation rate of c-kit gene among different age groups, different gender groups, different tumor size groups, and different mitotic image groups.

The diagnosis of gastrointestinal stromal tumor with multislice spiral CT is shown in Figure 4. It can be seen from the figure that when using virtual reality technology to process images with more texture information and images with less texture information, ACO and AACO can achieve better results, especially for images with more texture information, the effect is better, and the image clarity is higher, and the visual effect is better. At the same time, in terms of the continuity of the edge image, the continuity of SFLA-AACO edge image is slightly better than that of ACO and AACO edge image, because the edge image extracted by ACO and AACO has obvious breakpoints and discontinuous lines compared with SFLA-AACO edge image. The ideal image feature information can be obtained.

The CT test results of gastrointestinal stromal tumors are shown in Figure 5. Unfold different types of stomach nodules into a time series, and compare the smoothness of the time series to easily distinguish the difference between no sign, leaf sign, and glitch sign. The recursive graph algorithm comprehensively considers the chaos, nonstationarity, and periodicity of the gastric nodules boundary. At the same time, the algorithm in this paper has high specificity and low misdiagnosis rate, which avoids the interference of nonnodules to the doctor's diagnosis to a certain extent, and saves the doctor's diagnosis time. The algorithm is stable and reliable, does not depend on the overall gray value of the image, and has strong adaptability, which is conducive to the actual clinical application of gastric CAD.

### 4.2. Immunohistochemistry Results

The immunohistochemical composition of GISTs is shown in Table 4. The statistics are mainly based on the pathology reports of patients with gastrointestinal stromal tumors and liver metastases. According to my country's gastrointestinal stromal tumor diagnosis and treatment guidelines, it is the best plan to carry out genetic testing for patients, but patients who have undergone genetic testing in our hospital have few and incomplete data, so this case group was not accepted. In this proportion group, 46 cases (95.83%) were positive for CD117, 38 cases were positive for CD34 (79.17%), and 31 cases were positive for D0G1 (79.17%).

The immunohistochemical results of gastrointestinal stromal tumors are shown in Figure 6. The general properties of GIST patients can be divided into solid, cystic and cystic, of which 271 (86.0%), cystic 7 (2.2%), cystic solid 37 (11.8%), and the most common ones are the reality. The clinical manifestations of liver GISTs are mainly related to the size of tumor and the growth mode of tumor. Most patients have no obvious specific clinical symptoms and signs in the early stage of the disease. The more common clinical symptoms can be manifested as upper abdomen discomfort, abdominal distention, loss of appetite, etc., and the rare symptoms are dyspnea and nausea. When the tumor increases to a certain extent, when the surrounding tissues or organs are compressed, corresponding compression symptoms can be produced, such as anorexia, dyspepsia, nausea, vomiting, and other symptoms. In this group, 6 cases showed abdominal discomfort, 4 cases showed abdominal distention, 4 cases showed abdominal mass, 2 showed anorexia, and 8 patients were found by relevant examination.

The expression of PCNA in GIST and its relationship with clinicopathological factors are shown in Table 5. Among 51 GIST cases, 26 cases (50.9%) were positive for PCNA, of which 3 cases were negative in the very low-grade malignancy group; 5 cases (33.3%) were positively expressed in 15 cases in the low-grade malignancy group; among the 24 cases in the moderately malignant group, 14 cases (58.3%) were positively expressed; in the high-grade malignancy group, 7 cases (77.8%) were positively expressed. Biological soft tissue is not a single elastic body. The change of its strain has a greater impact on the stress. At the same time, there are also differences between loading stress and unloading stress. For small deformation model simulation, it is possible to use linear viscoelastic theory to solve it. However, for the large deformation simulation of the soft tissue model, the characteristics of the nonlinear viscoelastic body are more significant. Therefore, when establishing the model and determining the model parameters, the linear method is used to achieve this. Although the complexity of the model is simplified and the calculation efficiency of the model is improved, it reduces the accuracy and authenticity of the model.

The positive rates of CD117, CD34, and D0G1 in GIST are shown in Table 6. 223 patients were tested on CD117 and CD34. The number of positive cases was 214 and 198, respectively, and the positive rates were 96.96% and 84.75%, respectively. The mutation rate of c-kit gene in gastrointestinal stromal tumor tissue was 88.2% for spindle cell type, and the mutation rate of c-kit gene in gastrointestinal stromal tumor tissue was 60.0% for epithelial cell type. The mutation rate of C-suite gene between different tissue types of gastrointestinal stromal tumors is different, which is statistically significant (*p* = 0.002). Through comparison and analysis, it is known that the mutation rate of the spindle cell type c-kit genetic factor is higher than that of the epithelial cell type (*p* = 0.033) and higher than that of the mixed cell type (*p* = 0.006).

## 5. Conclusions

With the development of electronic technology and computer technology, the field of medical image utilization will continue to expand, and medical image processing technology will also attract more and more attention. CT images are more and more widely used in clinical diagnosis and treatment. This paper analyzes the application of contrast enhancement technology, wavelet transform technology, and rough set theory in CT image enhancement, compares their characteristics, and obtains a new algorithm of CT image processing. After segmentation, the regional image composed of lymph nodes, and blood vessels contain all the lymph nodes of the original stomach CT image. We need to extract lymph nodes from the regional image composed of lymph nodes and blood vessels. Because the outer boundary of lymph nodes is in the fat region, we can extract all the nonadhesive lymph nodes of the stomach CT image by using the boundary prior knowledge. At the same time, as a kind of sophisticated and complex equipment, CT equipment is extremely important to its scientific management and maintenance. The purpose of quality assurance is to ensure the normal operation of the equipment in use and the best performance to protect the interests of patients. In short, when confirming the diagnosis of GIST, we must pay attention to the tumor cell morphology, density, and cell arrangement and combine the results of immunohistochemical staining.

## Figures and Tables

**Figure 1:** Imaging appearance of gastrointestinal stromal tumor (picture source: http://alturl.com/nqqfw).

**Figure 2:** Ultrasound appearance of gastrointestinal stromal tumor (picture source: http://alturl.com/gq3at).

**Figure 3:** Main features of gastrointestinal stromal tumors (picture source: http://alturl.com/xtxed).

**Figure 4:** Diagnosis of gastrointestinal stromal tumor with multislice spiral CT (picture source: http://alturl.com/dcyf8).

**Figure 5:** CT test results of gastrointestinal stromal tumors (picture from http://alturl.com/wv8sv).

**Figure 6:** Immunohistochemical results of gastrointestinal stromal tumors (picture source: http://alturl.com/xd4fc).

**Table 1:** Comparison of detection time.

Number of experiments	Algorithm (s)	Traditional random forest (s)	AdaBoost algorithm (s)
1	5.01	7.49	20.87
2	5.34	7.74	21.01
3	4.95	7.32	20.58
Average value	5.10	7.55	20.82

**Table 2:** Multivariate COX regression analysis of postoperative survival rate of patients.

Influencing factors	*p* value	Relative risk	95% confidence interval
Tumor size	0.009	1.434	0.928∼5.221
Complete resection	0.005	1.213	0.385∼2.237
Mitotic count	0.003	0.059	0.009∼0.380
Ki-67 index	0.645	1.546	0.243∼9.850

**Table 3:** Multivariate analysis of risk factors in the abdominal and pelvic implant transfer group.

Variable	OR (95% CI)	*p* value
Size	3.744 (1.388–10.101)	0.009
Growth mode	1.249 (0.441–3.538)	0.675
Serosal invasion	1.090 (0.382–3.115)	0.872
Ascites	6.364 (1.295–31.273)	0.023

**Table 4:** Immunohistochemical composition ratio of GISTs.

Immunohistochemistry	Number of cases	Number of positive cases	Positive rate (%)
CD117	48	46	95.83
CD34	48	38	79.17
D0G1	32	31	96.88

**Table 5:** PCNA expression in GIST and its relationship with clinicopathological factors.

	Number of cases	PCNA positive	PCNA negative	*X* ^2^ value	*p* value
Male	19	9	10	0.153	*p* > 0.05
Female	32	17	15		
<45	16	8	8	0.009	*p* > 0.05
≥45	35	18	17		
Stomach	38	21	17	1.094	*p* > 0.05
Small intestine	13	5	8		

**Table 6:** The positive rate of CD117, CD34, and D0G1 in GIST.

Immunohistochemical	Number	Positive cases	Positive rate (%)
CD117	223	214	95.96
CD34	223	198	84.75
D0G1	34	34	100

## Data Availability

No data were used to support this study.
